# The Application of Artificial Neural Network Combined with Virtual Reality Technology in Environment Art Design

**DOI:** 10.1155/2022/7562167

**Published:** 2022-05-14

**Authors:** Lei Han, Li Gan

**Affiliations:** ^1^School of Art and Design, Shaoyang University, Shaoyang 422000, Hunan, China; ^2^School of Design, NingboTech University, Ningbo 315100, Zhejiang, China

## Abstract

Virtual reality is a computer technology that produces a simulated environment. It is completely immersive and gives users the viewpoint that they are somewhere else. In recent times, it has become a highly interactive and visualization tool that has gained interest among educators and scholars. Art learning is a teaching-learning approach that is dependent on learning “*through the arts*” and “*with the arts*;” it can be a procedure in which art develops the medium of teaching-learning and an important model in some subjects of the curriculum. In this work, we develop a grey wolf optimization with the residual network form of virtual reality application for environmental art learning (GWORN-EAL) technique. It aims to provide metacognitive actions to improve environmental art learning for young children or adults. The GWORN-EAL technique is mainly based on the stimulation of particular features of the target painting over a default image. The color palette of the recognized image of the Fauve painter was mapped to the target image using the Fauve vision of the painter and represented by vivid colors. For optimal hyperparameter tuning of the ResNet model, the GWO algorithm is employed. The experimental results indicated that the GWORN-EAL technique has accomplished effectual outcomes in several aspects. A brief experimental study highlighted the improvement of the GWORN-EAL technique compared to existing models.

## 1. Introduction

Jaron Lanier is credited with coining the phrase “Virtual Reality” in the 1970s. Virtual reality (VR) has become a useful tool for researching human perception from a psychological, social, philosophical, and cognitive standpoint [1]. To overcome this barrier, it uses simulation to simulate what it would be like to interact with the computer using the five senses. Some issues arise when combining software and hardware in the creation of virtual reality or virtual reality-related applications. It is possible that an artificial neural network (ANN) might be a helpful tool in addressing the myriad VR difficulties. Curve fitting, classification, and pattern recognition are only a few of the applications of ANNs. Before diving into the function of ANNs in virtual reality, it is crucial to understand how VR has evolved through time. When Ivan Sutherland published “The Ultimate Display,” people popularized the phrase “virtual reality [2].” In order to keep the **hardware malware detectors (HMDs)** connected to the mainframe, people built one. The first data glove was invented. They made VR communicable through soft body motions. As a result, they invented the term “VIDEOPLACE” to describe their projections onto walls [3]. Art galleries utilize it since it was the first VE (Virtual Environment) to be designed. Extending this notion, the CAVE system was created and further employed for data visualization, where it was exhibited in a room rather than on the HMD. After a couple decades of clunky HMDs, VR finally made it to the Android operating system. Virtual reality's progress hinges on its fundamental characteristics [4]. Immersion and interaction are two of VR's most valuable features. People have achieved true immersion when they are fully immersed in virtual reality. By moving one's body around in every possible way, one may accomplish interactivity. Additionally, sensory feedback and virtual worlds may be employed in virtual environments. The subject's sensory condition at a certain point in exposure is referred to as “sensory feedback” [5]. It is the interrelationships between the virtual items and the surrounding environment that provide meaning to the virtual world. In the realm of military rehabilitation, VR is being used to its fullest potential. Here, people will cover the basics of artificial neural networks, and how they may be used in virtual reality. In order to create such an app, the selection of a suitable algorithm is critical to success [6]. Due to the ANN's versatility and connection, it is employed in this study. As an example, gesture recognition employs probabilistic neural networks, whereas facial recognition employs the multilayer perceptron. An overview of ANN-related algorithms and their training functions is provided in this review article, as well as a discussion of how these algorithms aid with VR development and interface challenges [7]. In addition, it examines whether or not additional approaches, such as ANN, are required for a complete VR experience. Each neuron in the brain is connected to trillions of other neurons via trillions of other connections [8]. Each neuron fires either independently or collectively in order to accomplish a certain goal. Since all neurons have synapses connecting them, the connectionist model explains how neurons work perfectly. Since the network generated by the linkages was nonrecurrent, this model was unable to support learning. This constraint was addressed with the invention of the perceptron [9]. The fundamental unit of processing in a neural network, the perceptron, accepts input in the form of associative units to allow pattern recognition. Some characteristics are selected by these associative units according to their functions. Perceptrons were originally designed to be used in machines, but subsequently grew into programmes that created the groundwork for the development of neural networks [10]. The neural network has a built-in ability to learn and adapt to its surroundings. With this characteristic, it may be used in the context of pattern recognition. Another characteristic of ANNs is that they may develop connection patterns via error approximation. Their ability to generalise makes it easier to see patterns in the test data that are comparable [11]. Both guided and unguided learning are included here. One of the most important models is the multilayer perceptron, or feedforward net, which is followed by the radial basis function [12]. Approximations with weighted weights are nothing more than training algorithms that have been transformed into models. For benchmark purposes, all the data gathered should be considered. There are three groups in which each issue might be placed. This is a weight-changing training set. Training comes to an end with the use of a validation set. Improved generalisation is one of its primary goals [13]. As the validity error grows, the training process grinds to a standstill. Predictor pattern recognition is the primary purpose of the third set of tests, which is a testing set for generalisation. As a result, the Jacobian matrix is limited in its ability to quantify performance by looking at the mean or total squared errors [14]. Performance may be quantified in a variety of ways, the most common of which is the mean. A “one-of-a-kind” differentiating algorithm or mathematical index is what we mean when we talk about a performance metric. Let us look at an example to better understand how ANN algorithms might vary depending on the application. Learning is a laborious process, and no one knows how many layers of neurons there are in the brain. A second-order derivative may be used to offset these drawbacks. When the inaccuracy with regard to the weights is more than 2E2, the step size is adapted to go in the direction of the optimum weight update. ANN offers a variety of training strategies for tackling issues in both the computer and biological sciences. For example, there are three training methods for computed tomography (CT) pictures. It is possible to update weights and biases in the direction of the performance function's negative gradient using a gradient descent algorithm (GDA) [15]. Another option is an algorithm that modifies weights in the direction of a rapidly diminishing performance function. The third is the quasi-Newton algorithm, which takes advantage of the fact that a goal is present.

A global variable may be used to hurdle the function, and the sum of squares technique can be used to do so. Each method has several training functions and subalgorithms if the module demands a greater convergence speed or falls within the paradigm of an image pattern recognition issue, for instance, [16]. However, there are a few consequences to the function that is accessible. Under the aforementioned criteria, the former will demand a huge amount of storage space, while the latter will fail horribly on the issue of function approximation [17]. A metaheuristic approach is used by a few learning algorithms, but gradient descent is used by the majority. Using a global search technique and a more comprehensive answer, this method is more comprehensive. A new hybrid technique to solve these issues has been presented. IOPSO-BPA (Improved Opposition-based Particle Swarm Optimization-Backpropagation Algorithm) blends global metaheuristics with gradient-based techniques. After calculating the training time and accuracy for eight benchmark tasks, the proposed hybrid algorithm is then compared against BPA, iOPSO, and iOPSO-GA (Genetic Algorithm) [18]. There are fewer dispersion options for BPA, but it will take longer to get there. In the presence of' changeable beginning circumstances, IOPSP-BPA yields fewer dispersion solutions. Our discussion of artificial neural networks (ANN) and their various training procedures is over. People may expect to learn more about this in the next few parts.

Nonverbal communication, such as facial expressions, may convey a great deal of information. People's emotional states may be gleaned from this, and their behavior is easier to decipher. AR/VR may be used to assist consumers with chores such as verifying their identity online. The backpropagation approach is used to train the ANN by taking into account the user's audio, video, and picture inputs [19]. In addition to its vast range of uses in entertainment, it has a significant impact on rehabilitation. More and more studies have looked at using ANN in virtual reality headsets to create realistic facial expressions for autistic, ADHD, and schizophrenia patients in order to improve their social communication abilities. In addition to all of the aforementioned strategies, ANN is also up against some competition inside itself. For example, we compared the Convolutional Network (CN) and the multilayer perceptron (MLP) to recognize static faces in various expressions and found CNs to be superior to MLPs (despite the design of CNs being influenced by the MLPs). In the twenty first century, virtual reality (VR) has found numerous innovative uses in virtual showmanship, video conferencing, online messaging, and online video gaming, among other areas.

In a work of art, textures are mapped to screen space pixels by using a technique called “texture mapping [20].” Texture mapping is a common technique in 3D graphics, particularly when trying to create realistic-looking models. In order to draw an item, for example, people merely need to apply a photograph of the thing or an image texture that we created ourselves to a structure that is compatible with the object's geometry. Texture mapping, on the contrary, may guarantee that the polygon's texture changes as it is altered. People can use this method to apply several texture pictures to a model with a large surface area. When it comes to creating the desired look, people need to apply texture control technologies. On this basis, the roadway space topological connection is formed and the approach of modelling the roadway body and roadway node separately is used [21]. Interpolation processing algorithms are used to provide a seamless transition while crossing highways. After noise reduction, the point cloud includes a lot of duplicated information. Data may be reduced to a manageable size using uniform sampling. The high frequency of these outliers will have an impact on model optimization and rendering output in subsequent stages. These outliers are all related. Identifying and removing the outliers will help to prevent the aforementioned problem. It is impossible to immediately place a photograph on a model with highly irregular or complicated geometry, so the model loses a lot of its authenticity [22]. It reduces the quantity of point cloud data and speeds up data processing and modelling. The modelling accuracy will be lower if point cloud surface characteristics are lost during sampling, so be sure to verify the boundary. The texture picture may be rotated and zoomed in when facing a certain form. Yao and Xue-Feng integrate the application of artificial intelligence in environmental design, analyze the design works with wide influence, and discuss the value and significance of artificial intelligence in applied environmental design, as well as its possible future development trend. The development of artificial intelligence in environmental design, focusing on the exploratory research in landscape design and interior design, as well as the thinking and answers brought by relevant research [23]. Jiping Hai promotes the development of environmental art design towards intelligentization by discussing the status quo of the development of the intelligent space environment. In [24], the smart home space and environmental art design are analyzed, the development of environmental art design to be intelligent is promoted, and people are provided with a better quality living environment.

## 2. Materials and Methods

In this work, a novel GWORN-EAL technique has been developed for providing metacognitive actions to improve environmental art learning for young children or adults. The proposed GWORN-EAL technique involves three major components, namely, preprocessing, ResNet50, and GWO algorithm.

### 2.1. Preprocessing

An RGB to CIELAB conversion was utilized for transforming an input image to CIELAB color space, whereas the important process occurs. Afterward, an image equivalent to *a*^*∗*^ and *b*^*∗*^ channels was processed individually. Previously, the local color transfer procedure begins, and all the 2 frames are segmented by intensity utilizing a 3-level thresholding technique. Therefore, it contains 4 independent images, 2 equivalent to input and 2 to the target image.

### 2.2. CNN-Based ResNet50 Model

In this work, the CNN-based ResNet50 model is employed for environmental art learning. The CNN was famous in other NNs with its efficiency with image, speech, or audio signal input. It contains 3 important kinds of layers that are convolution, pooling, and FC layers. ResNet employs the residual block to solve the gradient vanishing and degradation issues determined in CNN. A residual block increases the network operation [1].

Particularly, the ResNet system has led to an outstanding performance in ImageNet classification competition. Consequently, it outperforms the balance with extra input of residual block, and result of remaining block can be demonstrated as follows:

(1) $$\begin{array}{c} y=F\left(x,W\right)+x, \end{array}$$

whereas *x*, *W*, and *y* imply the input, weight, and experimental outcome of the remaining block. ResNet is comprised of distinct remaining blocks whereas the convolution kernel size of the convolution layer is differed from one another. A conventional expansion of RestNet consists of RestNet101, RetNet18, and RestNet50 [2]. A layered structure of ResNet50 is presented in Figure 1. The feature attained by ResNet has network positioned in the FC layer to compute image classification. Therefore, the SM method is employed to classify images.

### 2.3. GWO-Based Hyperparameter Tuning Model

As a machine learning engineer designing a model, you choose and set hyperparameter values that your learning algorithm will use before the training of the model even begins. In this light, hyperparameters are said to be external to the model because the model cannot change its values during learning/training. “Hyperparameters are parameters whose values control the learning process and determine the values of model parameters that a learning algorithm ends up learning. The prefix ‘hyper_' suggests that they are ‘top-level' parameters that control the learning process and the model parameters that result from it.” To optimally adjust the hyperparameter [25] values of the ResNet50 model, the GWO algorithm has been applied. Lately, new Swarm Intelligence (SI) optimization technique named GWO was proposed by Mirjalili et al. [3]. Indeed, it is an inspired algorithm which speeds up social and hunting hierarchy of GW. For developing the social behavior of GW, it is categorized as 4, including alpha (*α*), beta (*β*), delta (*δ*), and omega (*ω*). *α* is considered as optimum solution employed as *β* and *δ*, respectively, and residual solution comes under *ω*. The first 3 fittest wolves named *α*, *β*, and *δ* are near the prey that helps *ω* to recognize the food in difficult areas. In the encircling stage, wolf improves the position of *β* or *δ* as shown below:

(2) $$\begin{array}{c} \overset{⟶}{D}=\left|\overset{⟶}{C}\cdot {\overset{⟶}{X}}_{p\left(t\right)}-\overset{⟶}{X}\left(t\right)\right|,\\ \overset{⟶}{X}\left(t+1\right)={\overset{⟶}{X}}_{p\left(t\right)}-\overset{⟶}{A}\cdot \overset{⟶}{D}, \end{array}$$

whereas *t* denotes the existing iteration, ${\overset{⟶}{X}}_{p\left(t\right)}$ designates the existing position of prey and $\overset{⟶}{X}\left(t\right)$ determines the existing position of wolf, $\overset{⟶}{D}$ shows the distance amongst prey and wolves, and coefficient vectors $\overset{⟶}{A}$ and $\overset{⟶}{C}$ are acquired in the arithmetical expression as follows:

(3) $$\begin{array}{c} \overset{⟶}{A}=2\overset{⟶}{a}\overset{⟶}{r_{1}}-\overset{⟶}{a},\\ \overset{⟶}{C}=2\overset{⟶}{r_{2}}, \end{array}$$

whereas $\overset{⟶}{r_{\text{l}}}$ and $\overset{⟶}{r_{2}}$ determine 2 vectors created from [0, 1] in arbitrary manner, and the element of $\overset{⟶}{a}$ is linearly decreased from 2 to 0 for all the iterations. Now, *α*, *β*, and *δ* are assumed to be positioned nearer to the position of prey. During the hunting process, top 3 are optimum solution and residual wolf *ω* is feasible for replacing based on first 3 optimum wolves. The wolf position is upgraded by using the following equation:

(4) $$\begin{array}{c} {\overset{⟶}{D}}_{\alpha }=\left|{\overset{⟶}{C}}_{1}\cdot \overset{⟶}{X}-\overset{⟶}{X}\right|, \end{array}$$

(5) $$\begin{array}{c} {\overset{⟶}{D}}_{\beta }=\left|{\overset{⟶}{C}}_{2}\cdot \overset{⟶}{X}-\overset{⟶}{X}\right|, \end{array}$$

(6) $$\begin{array}{c} {\overset{⟶}{D}}_{\delta }=\left|{\overset{⟶}{C}}_{3}\cdot \overset{⟶}{X}-\overset{⟶}{X}\right|, \end{array}$$

(7) $$\begin{array}{c} {\overset{⟶}{X}}_{1}={\overset{⟶}{X}}_{a}-{\overset{⟶}{A}}_{2}\cdot \left({\overset{⟶}{D}}_{\alpha }\right), \end{array}$$

(8) $$\begin{array}{c} {\overset{⟶}{X}}_{2}={\overset{⟶}{X}}_{\beta }-{\overset{⟶}{A}}_{2}\cdot \left({\overset{⟶}{D}}_{\beta }\right), \end{array}$$

(9) $$\begin{array}{c} {\overset{⟶}{X}}_{3}=\overset{⟶}{X}-\overset{⟶}{A}\cdot \left({\overset{⟶}{D}}_{\delta }\right), \end{array}$$

(10) $$\begin{array}{c} \overset{⟶}{X}\left(\text{t}+1\right)=\frac{\overset{⟶}{X_{1}}+\overset{⟶}{X}+\overset{⟶}{X_{3}}}{3}, \end{array}$$

whereas $\overset{⟶}{X_{\delta }}$ indicates the position of $\delta ,{\overset{⟶}{X}}_{\alpha }$ displays the position of $\alpha ,{\overset{⟶}{X}}_{\beta }$ denotes the position of $\beta ,\overset{⟶}{{\text{C}}_{1}},\overset{⟶}{{\text{C}}_{2}}$, and $\overset{⟶}{{\text{C}}_{3}}$ epitomize the vector produced in arbitrary manner, and $\overset{⟶}{X}$ represents the position of existing solution [4]. The precise distance amongst existing solution and *α*, *β*, and *δ* is estimated according to the above equation. Equations (7)–(10) evaluate the latter location of existing solution. Whereas *t* describes the amount of rounds of ${\overset{⟶}{A}}_{1},{\overset{⟶}{A}}_{2}$, and ${\overset{⟶}{A}}_{3}$ represented as the arbitrary vector. The step size of *ω* wolf performed afterward; *α*, *β*, and *δ* are shown in Equations (5)–(7), respectively. Next, the resultant position of *ω* wolfs has been evaluated according to the equations.

## 3. Result and Discussion

This section validates the experimental result analysis of the GWORN-EAL technique. The results are tested using the environmental images, collected on our own.  Figure 2 showcases the sample test image, and the corresponding art generated image is depicted in Figure 3.

The process of segmentation is accomplished on the sample test image to recognize the different element in the given image. Figure 3, thus generated, is further visualized through the application of grey wolf optimizer in the ResNet Model. The image quality assessment in the research article is carried out by the three assessment metrics mentioned below:

- Mean square error (MSE): “the MSE represents the cumulative squared error between the compressed and the original image, whereas PSNR represents a measure of the peak error”
- Root mean square error (RMSE): “RMSE is a frequently used measure of the differences between values (sample or population values) and is predicted by a model or an estimator and the values observed”
- Peak signal-to-noise ratio (PSNR): “PSNR is an engineering term for the ratio between the maximum possible power of a signal and the power of corrupting noise that affects the fidelity of its representation”

To highlight the enhanced outcomes of the GWORN-EAL technique, a detailed experimental result analysis is made in terms of MSE, RMSE, and PSNR, as illustrated in Table 1.

Figure 4 reports the MSE examination of the GWORN-EAL technique on distinct set of test images. The results show that the GWORN-EAL technique has resulted in effective values of MSE. For instance, in image 1, the GWORN-EAL technique has obtained lower MSE of 10.8600. In addition, in image 3, the GWORN-EAL system has gained minimum MSE of 8.0600. Similarly, on image 4, the GWORN-EAL approach has attained lesser MSE of 10.4000. Likewise, on image 5, the GWORN-EAL technique has obtained reduced MSE of 11.5500.

Figure 5 depicts the RMSE examination of the GWORN-EAL method on distinct set of test images. The results outperformed that the GWORN-EAL technique has resulted in effective values of RMSE. For instance, on image 1, the GWORN-EAL approach has gained decreased RMSE of 3.2955. Also, in image 3, the GWORN-EAL technique has obtained reduced RMSE of 2.8390. Likewise, in image 4, the GWORN-EAL system has reached minimal RMSE of 3.2249. Followed by, on image 5, the GWORN-EAL technique has obtained lower RMSE of 3.3985.

Finally, a brief PSNR inspection of the GWORN-EAL technique is performed using different test images, as illustrated in Figure 6. The proposed GWORN-EAL technique has resulted in increased values of PSNR under all images. For instance, with image 1, the GWORN-EAL technique has gained higher PSNR of 27.4142 dB. Also, with image 3, the GWORN-EAL approach has attained maximum PSNR of 30.0041 dB. Followed by, with image 5, the GWORN-EAL algorithm has reached superior PSNR of 26.8792 dB. From the abovementioned tables and figures, it is apparent that the GWORN-EAL technique has the ability to effectually convert the images into art images.

## 4. Conclusions

It is possible to create a simulated world using virtual reality technology (VR). It is an immersive experience that transports users to a different location. Educators and academics alike have taken notice of its transformation into a powerful interactive and visualization tool in recent years. As a teaching-learning technique, art-based learning relies on learning both “through” the arts and “with” the arts; it can also be a procedure in which the medium of teaching-learning is developed through the arts. Using the residual network for virtual reality in environmental art learning (GWORN-EAL) technique, we have developed a grey wolf optimization. It seeks to provide metacognitive tasks to promote the learning of environmental art for young children or adults. It is a great resource. Over a base image, the GWORN-EAL approach attempts to elicit specific elements of the target painting. The Fauve painter's vibrant color palette was used to map the target image to the recognized image of the Fauve painter. The GWO algorithm is used to optimise the ResNet model's hyperparameters. The results of the experiments showed that the GWORN-EAL method was effective in a number of ways. The GWORN-EAL method outperformed current models in a small-scale experiment. [26].

## Figures and Tables

**Figure 1:** Layered structure of ResNet50.

**Figure 2:** Sample input image.

**Figure 3:** Sample art generated output image.

**Figure 4:** MSE analysis of GWORN-EAL technique with distinct images.

**Figure 5:** RMSE analysis of GWORN-EAL technique with distinct images.

**Figure 6:** PSNR analysis of GWORN-EAL technique with distinct images.

**Table 1:** Result analysis of GWORN-EAL technique with different images.

Test images	MSE	RMSE	PSNR
Image 1	10.8600	3.2955	27.4142
Image 2	9.6800	3.1113	28.4133
Image 3	8.0600	2.8390	30.0041
Image 4	10.4000	3.2249	27.7901
Image 5	11.5500	3.3985	26.8792

## Data Availability

The data used to support the ﬁndings of this study are available from the corresponding author upon request.
